The article "Meta-Analysis of Effects of Nutritional Intervention Combined with Calcium Carbonate D3 Tablets on Bone Mineral Density, Bone Metabolism, and Curative Effect in Patients with Osteoporosis" was published in 2022. Journal: Contrast Media Mol Imaging.

# Meta-Analysis of Effects of Nutritional Intervention Combined with Calcium Carbonate D3 Tablets on Bone Mineral Density, Bone Metabolism, and Curative Effect in Patients with Osteoporosis

**DOI:** 10.1155/2022/3670007

**Published:** 2022-06-24

**Authors:** Hua Ni, Shuchen Zhang, Xiaowen Niu, Sha Dai

**Affiliations:** ^1^Nutrition Department, Shanghai Skin Disease Hospital, Shanghai 200443, China; ^2^Nutrition Department, Shanghai Putuo District T. C. M Hospital, Shanghai 200062, China

## Abstract

To investigate the changes in bone mineral density, bone metabolism, and efficacy of nutritional intervention combined with calcium carbonate D3 tablets in patients with osteoporosis, a RevMan 5.2 software meta-analysis was conducted in this study. According to the therapeutic direction of nutritional intervention combined with calcium carbonate D3 tablets for osteoporosis patients, relevant literature were searched in Wanfang Medical, CNKI, VIP, and PubMed literature databases at home and abroad. Keywords included bone mineral density, bone metabolism, blood calcium (Ca), blood phosphorus (P), osteocalcin (OC), bone mineral density (BMD), serum alkaline phosphatase (ALP), efficacy, osteoporosis, and nutritional intervention. Literature that met the criteria were deleted, and meta-analysis was performed using RevMan 5.2 software. The results indicate that a total of 10 Chinese literature were included. Compared with the monotherapy group, the clinical efficacy, osteocalcin, BMD, alkaline phosphatase, calcium, and phosphorus were significantly higher in the combination group (*P* < 0.05). Based on calcium carbonate D3, treatment combined with nutritional intervention can enhance the clinical efficacy, bone metabolism, and bone mineral density of patients with osteoporosis, and nutritional intervention combined with calcium carbonate D3 tablets is a feasible program to promote the recovery of patients with osteoporosis.

## 1. Introduction

Osteoporosis is a common metabolic orthopedic disease, which tends to occur in the elderly. 60-year-old women are a high-risk group of osteoporosis. With the aging of society becoming more serious, the incidence of osteoporosis is increasing year by year [1]. Patients with osteoporosis are often accompanied by symptoms of reduced bone mineral density and increased risk of fracture. Due to certain particularity of the disease, this kind of patients indirectly increases the treatment cycle and economic pressure [2]. Clinical treatment of osteoporosis are mainly calcium intake and regulate habits; nutrition intervention is the main idea osteoporosis clinical treatment, calcium carbonate D3 tablets are often chosen as calcium supplements, and the drug contains lots of vitamins and trace elements which help to improve the patient's bone metabolism and improve bone mineral density. In addition, bone melon extract, collagen, and calcitriol are all commonly used drugs for clinical nutritional intervention of osteoporosis, and their effectiveness has been recognized [3, 4].

Drugs in recent years have become the guide thinking of clinical treatment of osteoporosis, and studies have shown that calcium carbonate D3 tablets and other effective drug combination therapy of osteoporosis can enhance the clinical effect [5–14]. However, the conclusion has not been unified recognition. Therefore, the relevant clinical literature of nutritional intervention combined with calcium carbonate D3 tablets in screening patients with osteoporosis at home and abroad should be searched and deeply studied. To investigate the changes in bone mineral density, bone metabolism, and efficacy of nutritional intervention combined with calcium carbonate D3 tablets in patients with osteoporosis, the RevMan 5.2 software was used for meta-analysis on the selected literature.

## 2. Related Work

Osteoporosis is an age-related metabolic disease. It is a disease of the elderly and high-risk groups. It is a disease in which the metabolism of postmenopausal women will change with age, bone formation, and bone absorption. And endocrine function recession leads to abnormal secretion of thyroid hormone levels and indirectly increases calcitonin which reduces the content of serum calcium, eventually leading to increased bone resorption, and bone formation of bone absorption equilibrium is broken, The patient's bone mass was significantly reduced [15]. Medical studies have shown that nutrition absorption and lifestyle can affect the occurrence and development of osteoporosis, so timely and effective nutritional intervention has important guiding significance for improving clinical symptoms of osteoporosis and preventing osteoporosis [16].

Bone mineral density refers to bone mass per unit area or volume, which is an important reference standard for clinical diagnosis and efficacy evaluation of osteoporosis [17]. Wu et al. [18] pointed out that the content and metabolic level of calcium, phosphorus, and other microelements can affect bone mineral density and bone volume and help to improve the clinical symptoms of limb function, waist, and back function of patients with osteoporosis. This study result shows that on the basis of calcium carbonate D3 tablets treatment, the combined use of nutritional interventions for patients with a osteoporosis higher curative effect and the related parameters of bone metabolism and bone mineral density were obviously improved, and prompt nutritional intervention with calcium carbonate D3 tablets therapy is to enhance the clinical curative effect and promote the recovery of patients with osteoporosis and reliable solution. The main reason may be that the gumelon extract injection of compound in traditional Chinese medicine injection contains a variety of effective components, all of which can play a positive role in promoting cell growth and differentiation and regulating bone metabolism. For example, a variety of free amino acids in the extract are essential raw materials in the synthesis of bone inflammatory growth factors. Injection of more melon extract is a kind of active ingredients which can improve blood supply obstacles, help patients with local blood circulation obstacle of callus, and play an analgesic effect by inhibiting prostaglandin secretion; the most abundant polypeptide injection in the active ingredients can promote the body's fibroblast growth factor, BMP, and bone growth factor synthesis of source sex, and in turn affect the bone formation and absorption process; this kind of composition has a certain biological activity and can promote cell mitosis and differentiation process and thus enhance activity; soluble bone collagen can promote the cell at the same time; collagen protein, collagen, and osteocalcin can improve bone metabolism and maintain the bone resorption synthesis speed balance effect of relevant indicators. In addition, the active polypeptide components of this nutritional intervention injection have a synergistic effect with melon extract, which can promote the synthesis and secretion of the bone-derived growth factor, thus enhancing the positive effect of promoting bone growth and improving clinical symptoms of osteoporosis on the basis of the clinical effect of calcium carbonate D3 tablets [19]. Sethuraman and Marwaha [20] showed that calcitriol combined with traditional calcium supplement therapy can increase bone mineral density and relieve pain symptoms of patients with osteoporosis. Therefore, from the perspective of calcitriol, the mechanism of nutritional intervention with calcitriol may be as follows: solidified triol as vitamin D supplement can be transformed in the liver and effectively regulate calcium and phosphorus metabolism, while calcium and phosphorus metabolism participate in the process of the bone metabolism and maintain bone volume. Calcitriol can inhibit bone absorption and promote bone mineralization by regulating calcium and phosphorus metabolism. In addition, the symptoms of bone loss caused by abnormal secretion of parathyroid hormone in patients with vitamin D deficiency can be improved. In addition, calcitriol is an active vitamin D, which can promote calcium absorption and reduce bone loss without increasing tissue metabolic burden [21].

Therefore, there is still room for further improvement in the design idea of this study. In the follow-up study, the scope of literature retrieval should be further expanded to ensure the acquisition of enough literature samples and meta-analysis based on them, which has important guiding significance for obtaining higher quality information data and improving the reference value of meta-analysis results.

## 3. Proposed Methods

### 3.1. Literature Retrieval

The types of studies and experiments were randomized controlled trials (RCT). Keywords were bone density, bone metabolism, clinical efficacy, osteocalcin, nutritional intervention, calcium carbonate D3 tablets, calcium (Ca), Pi (P), osteocalcin (OC), bone mineral density (BMD), and alkaline phosphatase (ALP). We searched and screened literature in domestic and foreign literature databases such as VIP, CNKI, PubMed, and Wanfang Medical Science, and searched literature in line with the research direction and keywords for nearly 10 years. At the same time, reference information can be obtained by contacting authoritative experts in related fields, and information can be supplemented and modified by contacting authors when the results of the included literature are not clear or data are missing. The literature is searched and screened strictly according to the title and keywords, and the included literature is guaranteed to have the approval documents of relevant institutions. The literature included for the first time were read and those literature with obvious operational errors, repeated contents, and inconsistent methods were deleted. Then, the selected literature were used, and the RevMan 5.2 software was used for meta-analysis on the selected literature.

### 3.2. Literature Screening Criteria

Inclusion criteria include the following: single drug therapy with calcium carbonate D3 tablets, calcium carbonate D3 tablets combined with nutritional intervention program to treat osteoporosis; the selection of research objectives follows the principle of randomness, without setting nationality, age, gender, salary, race, and other screening conditions; the rate of loss to follow-up during the follow-up was less than 20%; hold the audit and approval documents of relevant institutions; publication time ≤ 6 years; complete original clinical data; there was no obvious error in the research operation; and there was no difference in other variables except the study sample size. Exclusion criteria include the following: review, meta, case report, and conference abstract; cell and animal basic experiments; does not conform to the research direction; and subjects with normal hearing and hearing impairment were not taken as research objects.

### 3.3. Literature Outcome Indicators

The literature outcome indicators are clinical efficacy, osteocalcin, bone mineral density, serum alkaline phosphatase, blood calcium, and blood phosphorus.

### 3.4. Quality Evaluation

The modified Jadad score scale was used to evaluate the quality of randomized controlled studies. The total score of the scale ranged from 1 to 7, with ≤3 as low quality and ≥4 as high quality.

### 3.5. Statistical Methods

The research data were input into RevMan 5.2 statistical software for analysis. The statistical data were represented by risk ratio (RR), and the analytical statistics were represented by weighted mean difference (WMD) or standard mean difference (SMD). All effect sizes were expressed with 95% confidence interval (CI). Heterogeneity between results of each study was tested by the chi-square test. When the heterogeneity between studies was *P* < 0.1 and *I*^2^ ≥ 50%, subgroup or sensitivity was used to analyze the source of this property. When the heterogeneity among the research studies met with the conditions of *P* > 0.1 and *I*^2^ < 50%, the heterogeneity had no statistical significance, and the fixed effect model was used for meta-analysis. When the source of heterogeneity is not clear, the random-effect model and descriptive analysis of obvious clinical and methodological heterogeneity are used in the analysis.

## 4. Results

### 4.1. Literature Retrieval Results and Characteristics

The Chinese and English literature submitted in accordance with the main direction, keywords, and screening criteria of this study were retrieved from Wanfang, CNKI, and PubMed. A total of 300 related literature were detected, and 10 Chinese literature were deleted and included.  Figure 1 shows the specific process of literature retrieval. A total of 7 high-quality literature and 3 low-quality literature were included in this study, and the evaluation results of the literature characteristics and quality level of the 10 literature are given in Table 1. It should be noted that A, B, C, D, E, and F represent clinical efficacy, osteocalcin, bone mineral density, serum alkaline phosphatase, blood calcium, and blood phosphorus, respectively. There was no significant publication bias in the 10 included articles, as shown in Figures 2 and 3.

### 4.2. Meta-Analysis of Clinical Efficacy of Nutritional Intervention Combined with Calcium Carbonate D3 Tablets in Patients with Osteoporosis

A total of 4 literature were included. The heterogeneity test showed that there was heterogeneity among the literature (*I*^2^ = 67.0%, *P* = 0.03), and the random-effect model was used for analysis. The efficacy of the combination group was significantly higher than that of the single drug group, and the difference was statistically significant after the combination of all studies (RR: 1.25, 95% CI: (1.16, 1.36), *P* < 0.00001). It is believed that nutritional intervention combined with calcium carbonate D3 tablets can improve the clinical efficacy of osteoporosis, as shown in Figures 4 and 5.

### 4.3. Meta-Analysis of Osteocalcin in Patients with Osteoporosis by Nutritional Intervention Combined with Calcium Carbonate D3 Tablets

A total of 5 literature were included, and the heterogeneity test showed that there was heterogeneity among literature (*I*^2^ = 95.0%, *P* < 0.00001). The random-effect model was used for analysis, and osteocalcin level in the combination group was significantly higher than that in the monotherapy group, with statistically significant differences between the combined studies (RR: −0.41, 95% CI: (−0.53, −0.30), *P* < 0.00001). It is thought that nutritional intervention combined with calcium carbonate D3 tablets can increase osteocalcin levels in osteoporosis, as shown in Figures 6 and 7.

### 4.4. Meta-Analysis of Nutritional Intervention Combined with Calcium Carbonate D3 Tablets on Bone Mineral Density in Patients with Osteoporosis

A total of 8 literature were included, and the heterogeneity test showed that there was heterogeneity among literature (*I*^2^ = 93.0%, *P* < 0.00001). The BMD of the combination group was significantly higher than that of the monotherapy group, and the difference was statistically significant (RR: 0.07, 95% CI: (0.06, 0.08), *P* < 0.00001). It is thought that nutritional intervention combined with calcium carbonate D3 tablets can increase bone mineral density levels in osteoporosis, as shown in Figures 8 and 9.

### 4.5. Meta-Analysis of Nutritional Intervention Combined with Calcium Carbonate D3 Tablets on Serum Alkaline Phosphatase in Patients with Osteoporosis

A total of 6 literature were included, and the heterogeneity test showed that there was heterogeneity among literature (*I*^2^ = 86.0%, *P* < 0.00001). The ALP in the combination group was significantly higher than that in the monotherapy group, and the difference was statistically significant (RR: 6.86, 95% CI: (5.45, 8.27), *P* < 0.00001). It is suggested that nutritional intervention combined with calcium carbonate D3 tablets can increase ALP levels in osteoporosis, as shown in Figures 10 and 11.

### 4.6. Meta-Analysis of Serum Calcium in Patients with Osteoporosis by Nutritional Intervention Combined with Calcium Carbonate D3 Tablets

A total of 6 literature were included, and the heterogeneity test showed that there was heterogeneity among literature (*I*^2^ = 99.0%, *P* < 0.00001). The random-effect model was used for analysis, and serum calcium in the combination group was significantly higher than that in the monotherapy group, with statistically significant differences between the combined studies (RR: 0.28, 95% CI: (0.26, 0.36), *P* < 0.00001). It is suggested that nutritional intervention combined with calcium carbonate D3 tablets can increase blood calcium levels in osteoporosis, as shown in Figures 12 and 13.

### 4.7. Meta-Analysis of Nutritional Intervention Combined with Calcium Carbonate D3 Tablets on Blood Phosphorus in Patients with Osteoporosis

A total of 6 literature were included, and the heterogeneity test showed that there was heterogeneity among literature (*I*^2^ = 96.0%, *P* < 0.00001). The randomized effect model was used for analysis, and blood phosphorus in the combination group was significantly higher than that in the monotherapy group, with statistically significant differences between the combined studies (RR: 0.09, 95% CI: (0.07, 0.10), *P* < 0.00001). It is suggested that nutritional intervention combined with calcium carbonate D3 tablets can increase blood phosphorus levels in osteoporosis, as shown in Figures 14 and 15.

## 5. Conclusions

In this study, a RevMan 5.2 software meta-analysis was conducted to investigate the changes in bone mineral density, bone metabolism, and efficacy of nutritional intervention combined with calcium carbonate D3 tablets in patients with osteoporosis. Nutritional intervention combined with calcium carbonate D3 in the treatment of patients with osteoporosis can improve clinical efficacy, bone mineral density, and bone metabolism, which is conducive to the recovery of patients with osteoporosis and has the feasibility of clinical promotion.

## Figures and Tables

**Figure 1:** Literature retrieval route map.

**Figure 2:** Overall literature bias plot.

**Figure 3:** Literature bias plots of each article.

**Figure 4:** Forest map of clinical efficacy.

**Figure 5:** Funnel plot of clinical efficacy.

**Figure 6:** Osteocalcin forest map.

**Figure 7:** Osteocalcin funnel diagram.

**Figure 8:** Forest map of bone density.

**Figure 9:** Funnel plot of bone mineral density.

**Figure 10:** Serum alkaline phosphatase forest map.

**Figure 11:** Funnel diagram of serum alkaline phosphatase.

**Figure 12:** Blood calcium forest map.

**Figure 13:** Blood calcium funnel diagram.

**Figure 14:** Blood phosphorus forest map.

**Figure 15:** Funnel plot of blood phosphorus.

**Table 1:** Literature quality characteristics.

Author	The year of publication	Outcome index	Quality score
Wang and Xu [5]	2011	BCD	4
Li et al. [6]	2021	ACEF	5
Zhang and Lin [7]	2011	AC	3
Dai et al. [8]	2018	ACDEF	6
Zhang et al. [9]	2018	BCDEF	6
Wang [10]	2016	ADEF	5
Zeng et al. [11]	2021	BCDEF	6
Yan et al. [12]	2021	BC	3
Zhao et al. [13]	2019	B	2
Liu [14]	2020	CDEF	5

## Data Availability

The data used to support the findings of this study are available from the corresponding author upon request.
